# Antimicrobial Drug-resistance Profile of *Vibrio Parahaemolyticus* isolated from Japanese Horse Mackerel (*Trachurus Japonicus*)

**DOI:** 10.14252/foodsafetyfscj.D-21-00001

**Published:** 2021-09-24

**Authors:** Tasturo Nishino, Hideki Suzuki, Shiro Mizumoto, Hirotaka Morinushi, Hiromi Nagaoka, Keiichi Goto, Shigeki Yamamoto

**Affiliations:** 1 Earth-Environmental Service Co., Ltd., 17 Kanda, Konyacho, Chiyoda-ku, Tokyo 101-0035, Japan.; 2 Shizuoka Institute of Environment and Hygiene, 232-1 Yainaba, Fujieda 426-0083, Japan.; 3 Section of Food Science, Department of Fisheries, School of Marine Science and Technology, Tokai University, 3-20-1 Orido, Shimizu-ku, Shizuoka 424-8610, Japan.; 4 Food Safety Commission of Japan, Akasaka Park Bldg. 22F, Akasaka 5-2-20, Minato-ku, Tokyo 107-6122, Japan.

**Keywords:** antimicrobial drug resistance, Japanese horse mackerel (*Trachurus japonicus*), *Vibrio parahaemolyticus*

## Abstract

This study aimed at investigating antimicrobial resistance (AMR) profile of *Vibrio parahaemolyticus (V. parahaemolyticus).* The bacteria were isolated from wild-caught and farmed Japanese horse mackerel (*Trachurus japonicus*), and examined for the antimicrobial drug resistance. Furthermore, the serotype, and the genes of thermostable direct hemolysin (*tdh*) and cholera toxin transcriptional activator (*toxR*) of the isolates were investigated by using a serotype testing kit and PCR method. Eighty-eight and 126 *V. parahaemolyticus* strains were isolated from wild-caught and farmed Japanese horse mackerel, respectively. Ten and 18 distinct serotypes were detected from wild-caught and farmed Japanese horse mackerel. All strains were negative for *tdh* genes but positive for *toxR* genes. Resistances to ampicillin (ABP) and to both ABP and fosfomycin (FOM) were observed in 54 and 23 strains from the wild-caught fish, while those resistant strains from farm fish were 112 and 7 strains. Multidrug-resistance to three or four drugs including ABP was observed in one or two strains from the wild-caught fish.

These results strongly suggest that the environmental exposure of antimicrobial drugs results in the spread of resistant genes in Japanese horse mackerel. This study highlights the need for monitoring the spread of resistance genes to the human intestinal flora as well as to other bacteria in the environment.

## 1. Introduction

Methicillin-resistant *Staphylococcus aureus*, vancomycin-resistant *Enterococcus* and multidrug-resistant *Pseudomonas aeruginosa* have become serious health problems as causative agents of medical-related infections in Japan. Problems of drug resistance such as the increased prevalence of multidrug-resistant and super multidrug-resistant tuberculosis are spreading throughout the world. Japanese government established the “National Action Plan on Antimicrobial Resistance (AMR)” in 2016 to continuously monitor the consumption of antimicrobial agents and drug-resistance development and to precisely identify various indicators of drug resistance in order to monitor emerging trends^1^^)^. Food Safety Commission of Japan (FSCJ) also established its action plan to implement until 2020 to promote and improve furthermore food safety risk assessment in relation to drug resistant bacteria. A systematic surveillance and monitoring system of drug resistant bacteria, specifically for the influence of drug resistant bacteria on human health through intake of seafoods, has not been established in the fisheries field^1^^)^. Several reports have been published about AMR profile of *Vibrio parahaemolyticus (V. parahaemolyticus)* isolated from fish, shellfish and seafoods in various countries^2^^,^^3^^,^^4^^,^^5^^,^^6^^,^^7^^,^^8^^,^^9^^,^^10^^,^^11^^,^^12^^)^. The accumulation of scientific knowledge and information are thus necessary for such assessments.

In the present study, we focus on the drug resistance of *V. parahaemolyticus* as a causative agent of food poisoning that has been linked to seafoods. In addition to the drug resistance, serotypes and pathogenic gene profile of *V. parahaemolyticus* isolated from wild-caught and farmed (in Shizuoka, Japan) Japanese horse mackerel (*Trachurus japonicus*) were examined.

## 2. Materials and Methods

### 2.1 Japanese Horse Mackerel

Twenty-four wild-caught Japanese horse mackerel were purchased at a retail store in Shizuoka, Japan, and 40 Japanese horse mackerel farmed in Shizuoka, Japan, were purchased from an aquaculture company (Shizuoka Fisheries Cooperatives Numazu Office). They were obtained from July to September 2016.

### 2.2 Isolation and Identification of *V. parahaemolyticus*

*V. parahaemolyticus* was isolated from the muscle (edible parts), gill and viscera collected from individual Japanese horse mackerel with scissors aseptically. Bacteria were isolated by a qualitative test method recommended by the National Institute of Health Sciences (http://www.nihs.go.jp/fhm/mmef/pdf/protocol/NIHSJ-06_ST4%20201607.pdf). The separation and identification processes are described briefly as follows. Each collected part was diluted 10-fold with alkaline peptone broth (Nissui Pharmaceutical, Co., Ltd., Tokyo Japan) and cultured at 35°C for 18 hours without shaking. A portion of the culture was then spread on CHROMagar (BD Japan, Tokyo, Japan). Vibrio culture medium, and typical light purple colonies were picked up as suspected colonies. Characterization and identification of isolates were performed using 1% NaCl-added TSI culture medium (Nissui Pharmaceutical, Co., Ltd.), 1% NaCl-added LIM culture medium (Nissui Pharmaceutical, Co., Ltd.), Nutrient Broth (BD Japan), 8% NaCl-added Nutrient Broth, 2% NaCl-added VP semi-solid medium (Eiken Chemical, Co., Ltd., Tokyo, Japan) and cytochrome oxidase test filter paper (Nissui Pharmaceutical, Co., Ltd.).

### 2.3 Serotyping

Serotypes O group and K were examined with *V. parahaemolyticus* typing immune sera, “Seiken” (Denka Company, Ltd., Tokyo, Japan).

### 2.4 Pathogenic Gene Test

DNA was extracted by the hot extraction method, and thermostable direct hemolysin (*tdh*) genes were identified by PCR^13^^)^. The primer set PVD-1 and PVD-2 (Takara Bio, Shiga, Japan) was used for *tdh* and the primer set constructed according to Kim et al^14^^)^ was for cholera toxin transcriptional activator gene (*toxR*). The *toxR* gene produces ToxR protein, which controls *tdh* gene expression^14,16)^.

### 2.5 Drug Resistance Test

Drug resistance tests were performed using the disc method (KB disc, Eiken Chemical, Co., Ltd.). Briefly, the test organism was grown at 37°C overnight in 1% NaCl-BHI broth (74 rpm). Cultured organism was diluted at turbidity of Mcfarland 0.5 by 1% NaCl-BHI, and 200 µl sample was cultured at 37°C overnight on Mueller Hinton II agar plate with discs. Discs of ampicillin (ABP) 10 µg/disc, fosfomycin (FOM) 50 µg/disc, tetracycline (TC) 30 µg/disc, and sulfamethoxazole/trimethoprim (ST) combination 23/75 µg/disc were used. Judgments were based on the criteria provided with the KB disc.

## 3. Results and Discussion

### 3.1 Isolation of *V. parahaemolyticus*

A total of 88 and 126 *V. parahaemolyticus* strains were isolated from the wild-caught and farmed Japanese horse mackerel, respectively (Table 1).

**Table 1.** Number of *V. parahaemolyticus* isolated from each part of wild-caught or farmed Japanese horse mackerel

Parts	Total number of fish samples	Number of fish samples contaminated with *V. parahaemolyticus* (%)	Number of isolates
Wild-caught			
Muscle	24	8 (33.3)	40
Gill	24	6 (25.0)	44
Viscera	24	3 (12.5)	4
Total			88
Farmed			
Muscle	40	0 (0.0)	0
Gill	40	15 (37.5)	78
Viscera	40	48 (17.5)	48
Total			126

### 3.2 Serotyping

Ten serotypes were detected in the isolates from the wild-caught mackerel. For the farmed mackerel, 18 serotypes were detected (Table 2).

**Table 2.** Serotypes of *Vibrio parahaemolyticus* isolated from wild-caught or farmed Japanese horse mackerel

Wild-caught		Farmed	
Serotype	Number of strains (%)	Serotype	Number of strains (%)
O2:KUT^1^^)^	30 (34.1)	O1:K32	35 (27.8)
O4:KUT	12 (13.6)	O3:KUT	20 (15.9)
O2:K3	8 (9.1)	O2:K28	17 (13.5)
O3:K45	7 (8.0)	O5:K17	14 (11.1)
OUT^2^^)^:KUT	7 (8.0)	O11:KUT	7 (5.6)
O3:K5	6 (6.8)	O4:K42	5 (4.0)
O3:KUT	6 (6.8)	O4:K9	4 (3.2)
O10:KUT	5 (5.7)	O10:K52	4 (3.2)
O2:K28	5 (5.7)	O1:K5	3 (2.4)
O4:K34	2 (2.3)	O1:KUT	3 (2.4)
		O3:K33	3 (2.4)
		O11:K36	3 (2.4)
		O2:KUT	2 (1.6)
		O4:KUT	2 (1.6)
		O3:K5	1 (0.8)
		O3:K57	1 (0.8)
		O6:K46	1 (0.8)
		O10:KUT	1 (0.8)
Total	88 (100.0)		126 (100.0)

^1)^ KUT: K untypeable

^2)^ OUT: O untypeable

O3:K6 strain, a pandemic strain of *V. parahaemolyticus*, was not isolated in this study, but serotype O1KUT and O2:K3, O3:K5, O3:KUT, O4:KUT, O5:K17, and OUT:KUT strains were isolated. Some researchers have reported that some isolates of these serotypes showed the same characteristics with the pandemic clone. In addition to the serotypes that we detected, O11:KUT, O4K42, O4K9 have been also postulated as pandemic strains^17^^,^^18^^,^^19^^,^^20^^)^.

### 3.3 Detection of Pathogenic Genes

None of the strains isolated were *tdh* gene-positive, while all strains were *toxR* gene-positive. The *toxR* gene has widely been used for identification of *V. parahaemolyticus*, and therefore, all the strains isolated in this study were judged to be *V. parahaemolyticus*^4^^)^.

Gene transfer from *tdh* gene-positive strains enables other bacteria to produce the toxin, i.e. integrative, and conjugative elements are self-transmissible modular mobile genetic elements integrated into a host genome that are passively propagated during chromosomal replication and cell division, and mediate the acquisition of complex new traits in bacteria^21^^)^. Therefore, it is presumed that gene transfer plays a role in *tdh* gene-negative *V. parahaemolyticus* acquiring the capability of producing the TDH toxin^15^^,^^16^^)^.

We were unable to isolate *tdh*-positive *V. parahaemolyticus*. Other studies have attempted to isolate *tdh*-positive strains from seafood and environmental samples. TDH-producing *V. parahaemolyticus* was previously isolated mainly from clams and oysters^22^^,^^23^^)^. It is supposed that the contamination rate of TDH-producing *V. parahaemolyticus* in fish might not be high in Japan, even though food poisoning associated with consumption of fish is caused by TDH-producing one.

### 3.4 Antimicrobial Drug Resistance

The resistance to ABP and to both ABP and FOM were observed in 54 and 23 strains, respectively. Wild-caught and farmed fish, in this study, had 112 and 7 strains, respectively. Multidrug resistance to three or four drugs including ABP was observed in one or two strains from the wild-caught fish (Table 3).

**Table 3.** Antimicrobial resistance profile of *Vibrio parahaemolyticus* isolated from wild-caught or farmed Japanese horse mackerel

	Wild-caught	Farmed
Antimicrobial drugs	Number of strains (%)	Number of strains (%)
ABP	54 (61.4)	112 (88.9)
FOM	1 (1.1)	0 (0.0)
ABP FOM	23 (26.1)	7 (5.6)
ABP TC ST	1 (1.1)	0 (0.0)
ABP FOM TC ST	2 (2.3)	0 (0.0)
Sensitive	7 (8.0)	7 (5.6)
Total	88 (100.0)	126 (100.0)

According to the statistics of sales amounts of antibiotics in 2019 reported by the Ministry of Agriculture, Forest and Fisheries^24^^)^, the amounts for fish in seawater were 22,610.8 kg of ABP, while TC of 9,598 kg and FOM of 319.1 kg were also reported. ST was not used for fish, but was used for human^25^^)^ and for livestock (pigs and chickens). The amounts of ST was not reported, but 44,389 kg of sulfamethoxazole and 10,183.2 kg of trimethoprim were used for livestock. Reasons of detection of antimicrobial resistance to ST are still unknown, but we supposed that the use of this drug in human and livestock might affect acquisition of resistance.

ABP resistance is most prevalent in our study, and other reports also showed ABP resistance is most prevalent in different places in the world including China and Korea^2^^,^^3^^,^^4^^,^^5^^,^^6^^,^^7^^,^^8^^,^^9^^,^^26^^)^.

Most of the resistance except for ABP was characterized by multidrug-resistant strains in the present study. Detection of multidrug resistant *V. parahaemolyticus* has also been reported in isolates from fish, shellfish, and/or seawater in Korea^2^^,^^3^^)^, Poland^4^^)^, China^6^^)^, and India^9^^)^. Multidrug-resistant pattern is different among these isolates, but some of these isolates are ABP, TC and ST resistant as observed in the present study. Multidrug resistance is considered a serious public health issue. A greater number of multidrug-resistant *V. parahaemolyticus* strains were isolated from wild-caught mackerel than farmed mackerel. It is supposed that wild-caught mackerel might be affected by environmental conditions of resistant-gene delivery to a greater extent than farmed fish.

Since resistance has been detected in various species of the genus *Vibrio*^10^^,^^11^^,^^12^^,^^27^^)^, it is possible that resistance genes have been transmitted throughout the genus. As such, drug-resistant *V. parahaemolyticus* may be involved in transmission of resistance genes to other bacteria in the environment or in the human intestinal flora, further emphasizing the importance of drug resistance to public health. Further study is necessary to clarify the origin of drug resistance genes to marine environment.
